The article "Anomaly detection in multivariate time series data using deep ensemble models" was retracted in 2025. Reasons: duplicate publication; overlap with earlier publications; suspected computer-generated content; citations of retracted work.

# Anomaly detection in multivariate time series data using deep ensemble models

**DOI:** 10.1371/journal.pone.0303890

**Published:** 2024-06-06

**Authors:** Amjad Iqbal, Rashid Amin, Faisal S. Alsubaei, Abdulrahman Alzahrani

**Affiliations:** 1 Department of Computer Science, University of Engineering and Technology, Taxila, Pakistan; 2 Department of Computer Science and Information Technology, University of Chakwal, Chakwal, Pakistan; 3 Department of Cybersecurity, College of Computer Science and Engineering, University of Jeddah, Jeddah, Saudi Arabia; 4 Department of Information System and Technology, College of Computer Science and Engineering, University of Jeddah, Jeddah, Saudi Arabia; Air University, PAKISTAN

## Abstract

Anomaly detection in time series data is essential for fraud detection and intrusion monitoring applications. However, it poses challenges due to data complexity and high dimensionality. Industrial applications struggle to process high-dimensional, complex data streams in real time despite existing solutions. This study introduces deep ensemble models to improve traditional time series analysis and anomaly detection methods. Recurrent Neural Networks (RNNs) and Long Short-Term Memory (LSTM) networks effectively handle variable-length sequences and capture long-term relationships. Convolutional Neural Networks (CNNs) are also investigated, especially for univariate or multivariate time series forecasting. The Transformer, an architecture based on Artificial Neural Networks (ANN), has demonstrated promising results in various applications, including time series prediction and anomaly detection. Graph Neural Networks (GNNs) identify time series anomalies by capturing temporal connections and interdependencies between periods, leveraging the underlying graph structure of time series data. A novel feature selection approach is proposed to address challenges posed by high-dimensional data, improving anomaly detection by selecting different or more critical features from the data. This approach outperforms previous techniques in several aspects. Overall, this research introduces state-of-the-art algorithms for anomaly detection in time series data, offering advancements in real-time processing and decision-making across various industrial sectors.

## Introduction

As technology advances, we can capture and store large volumes of organized time-based data, making time series study more significant. Time series forecasting and identifying anomalies are crucial data analytic tasks in finance, healthcare, and manufacturing with broad applications. Deep learning has developed a powerful implement for concentrating on these issues, exceeding previous techniques for efficiency. Time series data may be utilized for a variety of purposes, including classification [1, 2], clustering [3], forecasting [4], and outlier detection. Obtaining pertinent understandings from this data begins new study paths in various sectors. Forecasting a time series requires projecting future values based on historical data. The complicated and usually nonlinear dynamics in time series data make this project challenging. Anomaly detection aims to find odd or unexpected patterns in a time series. This task is difficult because of the complicated and frequently nonlinear connections inherent in time series data. Anomaly detection examines a time series for strange or unexpected tendencies. Anomalies may suggest issues or events that require attention, such as fraud, equipment malfunctions, or health risks. Time series anomaly detection is a critical problem with far-reaching implications in businesses as diverse as healthcare [5], security [6], and banking [7]. A pivotal study [8] established two categories of univariate time-series outliers. Although type I outliers happen independently, type II outliers might be linked to subsequent power fluctuations. Outlier detection and evaluation in time-series data is crucial for drawing meaningful inferences. If an expressive data analysis is to be performed, each outlier type must be adequately understood.

The article "Anomaly detection in multivariate time series data using deep ensemble models" was retracted in 2025. Reasons: duplicate publication; overlap with earlier publications; suspected computer-generated content; citations of retracted work.

This research looks at RNNs and (CNNs) as deep-learning models for predicting time series and anomaly detection. RNNs are particularly suited to time series forecasting since they can deal with subsequent data by retrieving previous insights and using them to guide future estimations. This research studies and compares the performance of multiple CNN and RNN variants, including LSTM [9], GNN, and Transformer against benchmark datasets. Two datasets can be utilized to assess the performance of the planned task. However, due to the severity and complexity of the benchmark credit card dataset, this concentrates on anomaly detection. Furthermore, we have seen multiple daily news broadcasts depicting credit card theft. Credit cards are a standard payment option for online and offline purchases [10]. Traditional anomaly detection approaches rely on statistical thresholds or heuristics, which might fail to detect minor anomalies. A more advanced anomaly detection method may be provided through deep learning models. Two well-known deep learning architectures effectively applied to this job are autoencoders and one-class classifiers. Anomalies are detected as data points that autoencoders cannot correctly rebuild as they learn to recreate the input data. Anomalies are discovered as data points that depart from a model of the typical behavior of the data using one-class classifiers. Older forecasting approaches, such as autoregressive integrated moving average (ARIMA) models, may fail to account for these complexities. On the other hand, deep learning models are great for time series forecasting due to their ability to discern detailed trends in data.

The article "Anomaly detection in multivariate time series data using deep ensemble models" was retracted in 2025. Reasons: duplicate publication; overlap with earlier publications; suspected computer-generated content; citations of retracted work.

Deep learning for time series forecasting and anomaly detection has various advantages [11]. In finance, machine learning techniques are utilized to anticipate stock prices, exchange rates for currencies, and numerous other financial variables. Deep learning algorithms in healthcare predict clinical outcomes, detect anomalies in medical imaging, and foresee prospective health issues. Deep learning algorithms detect machine flaws, optimize manufacturing processes, and increase industrial quality control. Deep learning has revolutionized time series forecasting and anomaly detection by introducing solid approaches for obtaining significant information from time series data. Unexpected patterns or occurrences in data streams may provide helpful information and aid in detecting conceivably risky or fraudulent behaviour. Instant inspection of highly complex [12] and complicated data streams [13] data flows is difficult. Many analytical [14], machine learning [15], and deep learning [16] methods have been successfully developed in recent years to address these issues. Deep learning is an even more effective time series forecasting and anomaly identification approach than previous techniques. Anomaly detection is the discovery of unusual or abnormal patterns in a time series. On the other hand, time series forecasting predicts probable outcomes of a time series based on current data. Deep learning algorithms can accurately capture complicated temporal linkages and erratic correlations in time series data, allowing them to estimate future values and identify abnormalities. Autoencoders or one-class classifiers are commonly used in deep learning anomaly detection. While learning to reconstruct the input data, autoencoders recognise anomalies as data points that cannot be correctly reproduced. One-class classifiers detect abnormalities as details that depart from a model of the data’s typical patterns. Various businesses have used these strategies to improve decision-making and problem-solving abilities. We should expect increasingly complex and accurate time series forecasting and anomaly detection solutions as deep learning progresses.

The most significant difficulty in time series anomaly identification is working with high-dimensional and intricate data. Previously, conventional statistical approaches like ARIMA [17] and exponential contouring [18] were used. Nonetheless, their ability to manage complicated data with various properties is limited. Latest techniques, such as isolation forests [19], autoencoder-based systems [20], and deep neural networks such as LSTM [21] and CNNs [16], have consistently detected abnormalities in high-dimensional complicated data. Conversely, these algorithms have drawbacks, exceptionally high processing costs, and a massive quantity of training data required. Another problem in time series anomaly detection is dealing with real-time high-volume data streams [22]. Typical batch-processing approaches are insufficient for real-time applications that require fast detection. As a result, new data analysis approaches have emerged, including live algorithms for recognising anomalies and sliding window-based [23].

The article "Anomaly detection in multivariate time series data using deep ensemble models" was retracted in 2025. Reasons: duplicate publication; overlap with earlier publications; suspected computer-generated content; citations of retracted work.

Finally, time series prediction and anomaly detection rely heavily on preprocessing. A few preprocessing methodologies, for example, standardization and element scaling, have been explored to expand the exhibition of profound learning models, and a clever procedure has been made. This work presents a measurable methodology for picking essential qualities from a dataset to address the constraints of high-layered sequencing information. Creating a data preprocessing strategy to improve anomaly detection accuracy is the primary contribution of this study. Coming up next is the paper’s prior commitment.

- A statistical strategy for selecting the most essential qualities from a dataset has been devised to handle high-dimensional data problems.
- Several deep learning models were tested by varying their parameters. With promising results, a Transformer-based network architecture has been proposed to identify time series data abnormalities.
- A GNN-based network architecture has been suggested and shown to discover time series data abnormalities.
- To increase system performance, an ensemble of multiple CNN and LSTM models has been proposed with an ensemble of several Transformer and GNN models.
- A thorough examination of conventional techniques for identifying time series anomalies across various circumstances and data sets.

The subsequent is the order of the paper. The related work section evaluates the relevant writings on anomaly detection. The proposed methodology section goes into great depth on the suggested technique for finding abnormalities. The next Section experiments presents extensive experimental results and observations from many models created by varying the network design and settings. Finaly the conclusion section summarises the study and emphasizes the valuable results.

## Related work

Researchers’ interest in time series anomaly identification and forecasting has recently peaked. Several new tactics have lately been implemented. Following is a comprehensive review of the most recently presented research on time series anomaly identification and forecasting utilizing deep learning. The authors [24] give a complete benchmark for assessing long-term time series forecasting models. The benchmark comprises datasets from various dynamic systems and real-world records, with trajectories ranging from 100 to 2000. The research also includes a benchmarking analysis employing traditional and cutting-edge models, including LSTM, DeepAR, NLinear, N-Hits, PatchTST, and LatentODE. The results provide exciting performance contrasts between various models, emphasizing the dataset-dependent aspect of model efficacy. The review offers a tailor-made inactive NLinear model, expanding DeepAR with an educational program learning stage. Both surpass their vanilla counterparts constantly.

The article "Anomaly detection in multivariate time series data using deep ensemble models" was retracted in 2025. Reasons: duplicate publication; overlap with earlier publications; suspected computer-generated content; citations of retracted work.

In this investigation, the authors [11] discuss various deep learning methods for anomaly detection. They proposed numerous deep learning and hybrid models for detecting outliers in multi-dimensional time series data. This study is essential and valuable due to the analysis of multiple models, the emphasis on real-world applications, and the emphasis on feature engineering. They also suggested a statistical method for dimensionality reduction in this paper. The investigation [25] looks at unsupervised anomaly detection (AD) algorithms for multivariate time series (MTS) from the Internet of Things (I). It lays the theoretical groundwork, examines existing AD approaches, and assesses 13 potential algorithms using two publicly accessible MTS datasets. Authors [26] also present a unique metaheuristic-based time series clustering approach for manufacturing abnormality identification, which addresses the issues of high computational complexity and changeable diversity in manufacturing time series data. The system collects cluster references from hierarchical and partitional clustering. It applies the extended compact genetic algorithm (ECGA) to determine optimal cluster centroid combinations using shape-based distance measurements and energetic temporal warping.

This work [27] analyses deep learning applications for anomaly detection in other sectors and explores numerous deep learning models utilizing various benchmark datasets. The research emphasizes the significance of carefully balancing performance, complexity, and interpretability when using ensemble deep learning. The study presented in the publication [28] comprehensively evaluates ensemble deep learning, an approach for improving machine learning performance. It delves into its theoretical basis, ensemble setups, usage, advantages, and disadvantages. The study also looks into deep learning-based approaches for detecting anomalies in multivariate time series (MTS) data, including RNNs, LSTM networks, and CNNs. Furthermore, [29] proposed a novel approach for detecting threats in real-time by combining stream analysis and machine learning. This architecture promotes less human-monitored circumstances, allowing for better identification of recognized and previously undiscovered threats and improved strike sorting and identifying anomalies processes. However, these findings declined considerably, as projected by the existing KDD dataset.

The article "Anomaly detection in multivariate time series data using deep ensemble models" was retracted in 2025. Reasons: duplicate publication; overlap with earlier publications; suspected computer-generated content; citations of retracted work.

The examined study [30] focuses on anomaly identification in streaming data. It proposes a novel method for evaluating live anomaly detection using entropy and Pearson correlation. Even though some operations were avoided owing to long batch processing times or data limits, big data broadcasting parts such as Kafka channels and Spark Streaming were employed to ensure scalability and applicability. The authors describe a novel semi-supervised recognition of anomalies framework built around neural procedures [31]. Because NPs are a robust probabilistic framework capable of describing function distributions, they are perfect for anomaly detection applications. The study methodology employs labelled and unlabeled data to calculate the range of standard patterns semi-supervised using NP flexibility. The conceptual system successfully identifies anomalies by learning a distribution across usual patterns and finding data that differ considerably from this pattern.

The study [32] present a time-series anomaly identification approach based on Transformer models and 1D CNNs. The TAD-STCNN approach extracts global temporal linkages and latent representations from time-series data, while a stack of 1D CNNs recovers high-level features and regional temporal trends. An anomaly detection component is needed to compute anomaly scores. The article [33] introduces a unique hybrid machine learning (HML) technique for identifying anomalies in MTS data. The suggested HML-MTSAD technique combines two complementary anomaly identification methods: physics-motivated KPIs and an unsupervised variational autoencoder (VAE) with LSTM layers. The KPIs gather expert data on the quality of MTS data. Nevertheless, the VAE-LSTM model draws latent models from data to detect abnormalities that the KPIs may miss.

The authors [34] introduce an innovative unsupervised identification of anomalies technique for multivariate time series (MTS) data based on self-learning neural networks known as generative adversarial networks (GANs). The DVGCRN paradigm incorporates spatial and temporal dependency in MTS data by merging deep variational inference with graph convolutional recurrent networks. Despite [35] concerns with computer complexity and hyperparameter adjustment, the investigation shows that this strategy dramatically improves anomaly identification performance in MTS data. The STAD-GAN architecture converts the given MTS into a latent model, subsequently fed into a deep neural network classifier. The system utilizes A self-training strategy, in which a teacher model provides pseudo-labels for unlabeled data, which is then used to train another student model.

The article "Anomaly detection in multivariate time series data using deep ensemble models" was retracted in 2025. Reasons: duplicate publication; overlap with earlier publications; suspected computer-generated content; citations of retracted work.

Combining numerous models, deep ensemble models increase effectiveness and give a more reliable conclusion. Their ability to collect varied patterns and correlations in time series data considerably improves their capacity to detect anomalies. Deep learning techniques like recurrent neural networks and augmented short-term memory networks may detect longitudinal associations and intricate patterns in time series data. Deep ensemble modeling of cognitive processes improved the interpretability of previously found anomalies and novel variables. However, challenges like a lack of labeled deviant data for training continue to exist, necessitating innovative approaches such as semi-supervised learning or artificial data synthesis strategies.

## Proposed methodology

The research uses machine and deep learning to focus on dataset preparation, preprocessing, and anomaly identification. It entails producing or extracting datasets to determine the region of interest and utilizing various anomaly detection algorithms. Deep learning algorithms such as CNN, LSTM, CNN-LSTM-Ensembled, DAGM, Transformer, GNN, and hybrid combinations are used in the suggested technique. Patterns, correlations, and anomalies in time series data are captured systematically. The review process guarantees that the optimal model is utilised for each assignment and gives valuable information about each method’s performance. The proposed method exhibits deep learning capacity in time series forecasting and anomaly detection issues, providing a versatile and effective solution for various applications. Fig 1 displays the entire planned procedure.

**Fig 1:** The proposed work generic workflow.

The investigation will be conducted employing the strategies depicted in Fig 2. These strategies are isolated into numerous crucial stages, and each step’s tasks are completed.

**Fig 2:** A detailed overview of the proposed anomaly detection methodology.

### A. Data acquisition

The primary stage is to gather time series information from demonstrated sources. The obtained information has now been sent to the framework, where it will be mined and investigated. This is the most crucial stage of the time series anomaly detection method.

The article "Anomaly detection in multivariate time series data using deep ensemble models" was retracted in 2025. Reasons: duplicate publication; overlap with earlier publications; suspected computer-generated content; citations of retracted work.

### B. Exploratory data analysis

Researchers utilise exploratory data analysis (EDA) to inspect and dissect informational collections, generally incorporated with information representation apparatuses. This empowers clients to control information sources more effectively to obtain wanted results, making finding designs, distinguishing abnormalities, testing speculations, and approving suppositions more straightforward. Prior to displaying, EDA investigates everything the information can say to us. It isn’t easy to distinguish essential data elements when viewing a single spreadsheet column or the entire spreadsheet. Fundamental insights, which can be tedious, complex, and scary, may be helped by exploratory information examination methods.

### C. Data preprocessing

A crucial step in looking into time series anomalies is preparing the data. Data become increasingly chaotic as a result of time series repetition and inconsistency. Information standardisation utilises information preprocessing as a separating approach. Normalisation, cleaning, timestamping, and occasional pattern disintegration are essential for information arrangement. This activity involves completing numerous steps to obtain the files in the correct structure. Fig 3 shows the information planning stages. As found in Fig 3, we first gather the dataset from the benchmark, then, at that point, run some preprocessing, clean information methodology, and evaluate assuming the information is in a sort of time series.

**Fig 3:** Different data preprocessing phases/steps.

### D. Feature extraction/ dimensionality reduction

Dimension diminution is essential for breaking down substantial volumes of raw data into convenient groups. Accordingly, handling increments is more successful. The different factors inside these broad data sets are essential, and understanding them requires enormous figuring power. This includes extraction, extricating the finest attributes from massive datasets by choosing and joining factors and lessening information size. These parts are simple to use and effectively transmit data. The statistical approach, principal component analysis (PCA), linear discriminant analysis (LDA), and TSNE are ways of distinguishing elements of data and decreasing dimensionality.

We introduce an optimal statistical measure for picking different or more significant components from a dataset to overcome the limits of high-dimensional arranging data. The recommended method determines the main characteristics, improving grouping results over other predominant qualities from publically accessible laid-out benchmark datasets. The methodology is like grouping arrangements that don’t require configuration. In numerous ways, it is desirable over the ongoing grouping. Also, the proposed strategy is direct, fast, and dependable. Moreover, it is remarkable, with a low expectation to learn and adapt. The accompanying methodologies decide on highlights that might segregate between different parts.

The article "Anomaly detection in multivariate time series data using deep ensemble models" was retracted in 2025. Reasons: duplicate publication; overlap with earlier publications; suspected computer-generated content; citations of retracted work.

When using this technique, a data collection of n classes can be exemplified by a matrix nm, wherever n is the number of classes and m is the number of features. To implement this technique, evaluate the mean and variance of every data class column by column. This will outcome in a mean vector for each class. Each class variance is processed as a result. To find measurably immense qualities that assist with separating isolated gatherings, we want to ascertain the typical distances, everything being equal, segment by section. For each set of classes (e.g., p and q), a standard distance vector is created utilizing the measurement given in Condition.

#### 1. Comparison with optimal statistical methods and without optimal statistical methods

The main aim of proposing a statistical method is to overcome high dimensionality issues and use only prominent and relevant features. As we have introduced this method for feature selection, no previous work should be compared with this method.

Table 1 shows the result of the optimal statistical method on different datasets. A positive "Diff_Recall" indicates that the model’s recall improves by adding optimal statistical methods, which might imply that these approaches aid in successfully catching positive cases, particularly in minority classes. A significant "Diff_FPR" indicates that statistical approaches improve the model’s false positive rate, implying a trade-off between sensitivity and specificity. Overall, examining these discrepancies gives valuable insights into the influence of statistical approaches on model performance, which helps decision-makers select and use appropriate techniques for classification tasks.

**Table 1:** Comparison of results with and without optimal statistical method.

Classifier	Dataset	Recall_WOSM	Recall	Diff_Recall	FPR_WOSM	FPR	Diff_FPR
CNN	Credit Card Fraud Detection	0.7674	0.8602	0.0928	0.7647	0.8602	0.0955
LSTM	Credit Card Fraud Detection	0.7941	0.8529	0.0588	0.7941	0.8529	0.0588
CNN-LSTM-Ensembled	Credit Card Fraud Detection	0.7867	0.8235	0.0368	0.7867	0.8235	0.0368
CNN	Credit Card Fraud Detection2023	0.9995	0.9995	0.0000	0.9995	0.9995	0.0000
LSTM	Credit Card Fraud Detection2023	0.9995	0.9994	-0.0001	0.9995	0.9994	-0.0001
CNN-LSTM-Ensembled	Credit Card Fraud Detection2023	0.9996	0.9997	0.0001	0.9996	0.9997	0.0001
Transformer	Credit Card Fraud Detection	0.8014	0.8308	0.0294	0.8014	0.8308	0.0294
GNN	Credit Card Fraud Detection	1.0000	1.0000	0.0000	1.0000	1.0000	0.0000
Transformer-GNN-Ensembled	Credit Card Fraud Detection	1.0000	1.0000	0.0000	0.8308	0.8529	0.0221
Transformer	Credit Card Fraud Detection2023	0.9996	0.9996	0.0000	0.9996	0.9996	0.0000
GNN	Credit Card Fraud Detection2023	1.0000	1.0000	0.0000	1.0000	1.0000	0.0000
Transformer-GNN-Ensembled	Credit Card Fraud Detection2023	0.9996	0.9996	0.0000	0.9996	0.9996	0.0000
DAGMM	Credit Card Fraud Detection	0.7238	0.7047	-0.0191	0.0145	0.0155	0.0010
DAGMM	Credit Card Fraud Detection2023	0.0851	0.0546	-0.0305	0.0169	0.0455	0.0286

The article "Anomaly detection in multivariate time series data using deep ensemble models" was retracted in 2025. Reasons: duplicate publication; overlap with earlier publications; suspected computer-generated content; citations of retracted work.

#### 2. Optimal statistical method

The suggested optimal statistical technique for feature selection is a unique approach to anomaly detection that has the potential to increase detection accuracy dramatically. It tries to minimize data dimensionality, lowering the danger of overfitting and enhancing the generalizability of anomaly detection models. The method also improves model performance by prioritising the most informative characteristics and removing redundant or unnecessary ones. This guarantees that anomaly detection models’ characteristics are highly discriminative, increasing anomaly identification accuracy. Statistical feature selection approaches naturally resist noise and outliers, emphasising characteristics with strong correlations to the target variable while limiting the effect of noisy or irrelevant information. This increases the resilience of anomaly detection models while decreasing false positive and false negative rates.

This transparency boosts trust in the feature selection process and makes model predictions easier to comprehend, allowing domain experts to understand better and confirm the results. The adaptable technique may be used in various fields outside anomaly detection, such as financial fraud detection, healthcare monitoring, and industrial process management. Overall, the suggested statistical technique for feature selection can considerably improve anomaly detection accuracy by allowing for more efficient data utilization, model performance, and interpretability.

Compared to existing methodologies, the suggested feature selection method offers numerous advantages. To begin with, it does not alter the prototype meanings of the attributes. The system then chooses attributes based on their statistical importance. Third, it succeeds or even improves categorisation performance. Fourth, the approach is straightforward, quick, simple, and computationally competent. Finally, it avoids the plague of dimension.

The article "Anomaly detection in multivariate time series data using deep ensemble models" was retracted in 2025. Reasons: duplicate publication; overlap with earlier publications; suspected computer-generated content; citations of retracted work.

### E. Deep learning-based classifiers

The emphasis will be on discovering and performing repetitious brain networks for layout purposes like LSTM, CNN 1D, outfits of LSTM, CNN, GNN, and Transformer, and gatherings of GNN, Transformer, and DAGMM throughout this stage. LSTM units are meticulously placed near the LSTM organisation’s information and outcome layers. For some applications, this method may discriminate between short- and long-haul circumstances without additional equipment. Peephole connections between internal partitions and gates in the same cell can also be used to test the performance of cutting-edge LSTM design. Deep LSTM RNNs (DNNs) contribute to developing more robust speech recognition algorithms. It is fundamental to dissipate boundaries over different layers while consolidating a profound LSTM CNN with an ordinary LSTM to develop settings further. This work will employ DAGMM algorithms with optimal and finely tuned parameters and LSTM, CNN, GNN, Transformer, and their ensembled models.

#### 1. LSTM

The LSTM kind of RNN was made to forestall lessening varieties in RNNs. LSTMs have been utilized in different explorations to distinguish and conjecture charge card peculiarities. LSTM models determine how to perceive major patterns and connections in charge card exchange information, which they can then use to foresee future exchanges. The LSTM stepwise method is depicted graphically in Fig 4. The critical element of the LSTM structure is the memory block known as the LSTM unit [36]. It comprises four feedforward brain structures with distinct details and outcome levels. They disregard the truth that information and result doors are three of the four feedforward brain networks answerable for data sifting. Possible memory, the fourth brain organization, creates new data about the possibility of being put away in memory.

**Fig 4:** LSTM network architecture for the proposed work.

LSTM networks are an effective method for detecting anomalies in time series data. They can successfully simulate complicated temporal patterns, enabling the identification of abnormalities over long periods. LSTMs also include memory cells that can store information over time, allowing them to recall previous observations and detect anomalies based on contextual information. They can handle variable-length sequences, making them adaptable to various time series datasets without needing fixed-length inputs. LSTMs can simulate nonlinear interactions between data points, allowing them to discover abnormalities in complex and dynamic situations. Feature extraction is automated during training, which eliminates the need for human feature engineering. LSTMs resist noise and missing data, which allows them to perform well in noisy or incomplete time series datasets. This resilience improves their capacity to detect abnormalities properly in real-world circumstances where data is contaminated or missing. Overall, LSTMs are an effective method for detecting anomalies in time series data.

The article "Anomaly detection in multivariate time series data using deep ensemble models" was retracted in 2025. Reasons: duplicate publication; overlap with earlier publications; suspected computer-generated content; citations of retracted work.

#### 2. Deep autoencoding gaussian mixture model (DAGMM)

DAGMM is a powerful unsupervised learning technique that detects high-dimensional, particularly time series data abnormalities. Merging deep autoencoder networks with a Gaussian Mixture Model (GMM) predicts regular variation in data, including anomalies. The GMM indicates the chance dissemination of the encoded data, whereas the autoencoder preserves the input data’s fundamental makeup and features. Looking for cases with a moderately low likelihood thickness yields irregularities. The proposed study uses DAGMM for oddity identification in the time series area, where finding strange examples and takeoffs from standard behaviour methods is basic [37]. The engineering chart of the model portrays its essential parts, which incorporate the encoder, which packs input information into a lower-layered dormant space; the GMM layer, which recreates the typical way of behaving; and the decoder, which plays information. DAGMM provides a solid way to deal with irregularities in opportunity series information, adding to the strategy’s general gauging and oddity location arrangement. Fig 5 shows an itemised outline of DAGMM.

**Fig 5:** Deep autoencoding gaussian mixture model architecture for the proposed work.

#### 3. Ensembled model

Ensembling is a deep learning approach that might be utilised by combining various models for different purposes like NLP, recognition of images, and time series. It blends multiple models with fluctuating qualities and weaknesses to conquer requirements and convey more exact projections [28]. A group can be shaped by averaging conjectures, weighting expectations given execution, or utlizing progressed methods like stowing, helping, or stacking. Profound learning strategies, including gathering learning with a self-consideration approach, make up for connections between information that group learning can’t remember. Bootstrap Amassing, helping, and stacking are well-known methods. Fig 6 portrays the module outline containing test affiliation learning and a coordinated discovery organisation.

**Fig 6:** Deep learning ensemble model architecture for the proposed work.

Bagging is the most common way of preparing various runs of similar model with different sorts of organising information and amassing their appraisals. Boosting entails training several weak models in perpetuity, with each succeeding model focused on examples erroneously identified by earlier models. Stacking entails building numerous models on comparable data and using a meta-model to offer the final forecast based on the results of the individual models. Ensemble models increase the ability of deep learning models when handling complicated and high-dimensional data. They are, in any case, computationally exorbitant and require cautious tweaking of hyperparameters to accomplish the best outcomes.

The article "Anomaly detection in multivariate time series data using deep ensemble models" was retracted in 2025. Reasons: duplicate publication; overlap with earlier publications; suspected computer-generated content; citations of retracted work.

#### 4. Deep CNN

Deep CNNs’ Fig 7 design has been shown to detect complicated correlations and relationships in successive data, which makes them excellent for time series forecasting applications. Their architecture learns hierarchical characteristics, which allows them to uncover patterns at different levels of abstraction [38]. The suggested method handles sequential time series data with varied properties, capturing multiple scales of local patterns using 1D convolution layers and down-sampling spatial dimensions with the maximum pooling layers. Dropout layers help to prevent overfitting, while batch normalisation keeps activation stable. After that, the output is connected to thick layers for further feature processing. Deep CNNs effectively detect local patterns in time series data, where local trends are critical for precise forecasting. Their construction is resistant to changes in time, making it appropriate for recording temporal dynamics.

**Fig 7:** Deep CNN network architecture for the proposed work.

#### 5. Transformer

The Transformer Fig 8 is an ANN design that has exhibited tremendous outcomes in different applications, for example, regular language handling, time series determining, and peculiarity location [32]. It outperforms recurrent neural networks like LSTMs in terms of parallelisation and long-term dependency management. The Transformer model might figure out how to recognise patterns and anomalies in Mastercard exchange records over the long haul, considering more exact expectations regarding future exchanges. It is a grouping-to-succession network that relies upon consideration procedures and has beaten other RNN-based models in irregularity discovery. The Transformer is partitioned into two sections: an encoder and a decoder, each with subnetworks and remaining associations. Its viability in distinguishing abnormalities is extraordinary.

**Fig 8:** Transformer network architecture for the proposed work.

#### 6. Graph neural networks (GNNs)

They may be used to discover time series anomalies by recording temporal connections and links among specific times. GNNs use time series data’s underlying graph structure, with each node representing a time point and edges expressing temporal dependence. They move data about the graph, looking for patterns and anomalies based on temporal relationships within time series. This method helps find deviations from expected temporal relationships [39]. Graph Convolutional Layers capture temporal correlations and extract characteristics from the temporal graph. The Readout Layer gathers data to generate a graph-level representation. Fully Connected Layers then assess the data, and the final output layer assigns an anomaly score to each time point. Anomaly detection is performed by establishing a threshold for anomaly scores and reporting occurrences that exceed the threshold as anomalies. GNNs give a helpful perspective to the proposed method by explicitly modelling the temporal relationships in time series data, boosting the ability to detect abnormal patterns that evolve. GNNs are deep learning networks that deal with material with intrinsic graph patterns, as seen in Fig 9.

The article "Anomaly detection in multivariate time series data using deep ensemble models" was retracted in 2025. Reasons: duplicate publication; overlap with earlier publications; suspected computer-generated content; citations of retracted work.

**Fig 9:** GNN network architecture for the proposed work.

At this stage, it is critical to predict abnormalities based on the data that comes in. Numerous method sequences could be required for the procedures to expand. The program facilitates the identification of anomalies and examines the consequences of receiving unusual data. Fig 10 illustrates the suggested solution’s entire flow diagram.

**Fig 10:** The proposed work’s detailed system block diagram.

### F. Anomaly detection

At this level, predicting abnormalities based on incoming data is critical. Numerous method cycles may be required for the methods to get more complex. It enhances anomaly detection accuracy. Improper data is sent back to the program, which assesses the results.

## Experiments

This investigation sought to evaluate the effectiveness of deep learning systems in identifying and forecasting credit card abnormalities. Deep learning algorithms were developed utlizing a massive dataset of credit card transactions, and their accuracy in detecting anomalies in real-time transactions, credit card usage patterns, and merchant transactions was tested.

### A. Experimental setup

The deciding and peculiarity acknowledgement preliminary game plan will integrate the up-to-date Python or Jupyter Diary frames, an AMD Radeon R7 M640 delineations card, Windows 10, an Intel(R) Center i7-4510U PC processor @ 2.00GHz 2.60GHz, and 16GB of Hammer. The technique will be taken a stab at using benchmark datasets. The objective is to cultivate a trustworthy system for recognising various issues using CNNs, which have recently been used to acknowledge Mastercard irregularities. CNNs are especially fitting for picture affirmation applications, yet they may similarly be used to see plans in undeniable data. CNNs may be ready on a dataset of Mastercard trades and, a short time later, used to perceive programs that are hailing inconsistencies in logical transactions, showing their precision and responsiveness.

The article "Anomaly detection in multivariate time series data using deep ensemble models" was retracted in 2025. Reasons: duplicate publication; overlap with earlier publications; suspected computer-generated content; citations of retracted work.

Deep learning calculations have been created to gauge future charge card exchanges, including use and misrepresentation risk. This study used the LSTM network, CNN, GNN, transformer DAGMM, and ensembled models to identify fraud. The model was evaluated utilizing precision, review, and F1-score measures, affirming its ability to foresee extortion accurately. As per the information, profound learning might distinguish and show Visa inconsistencies with high exactness, accuracy, review, F1-Score, MSE, and R2 Score.

### B. Dataset

The Numenta Anomaly Benchmark (NAB) is a dataset [40] that utilises over 50 labelled real-world and artificial time series data files for real-time anomaly detection algorithm benchmarking. It contains AWS server stats, Twitter level, ad click analytics and traffic statistics. The dataset consists of a scoring method favouring early detection while penalising late or incorrect outcomes and recognising online learning. NAB is a helpful resource for academics and developers working on anomaly detection algorithms since it provides a standard dataset and a scoring method for evaluating the performance of algorithms. Its primary characteristics include real-world data, labelled anomalies, online learning, and the fact that it is open-source. The following parts give information on the actual fraud detection for the credit card datasets involved in this study.

#### 1. Credit card fraud detection dataset

Credit card fraud detection algorithms [41] are often utilised in machine learning and data science. Attributes in the dataset include time, amount, class, and class prevalence. The information gathered from European credit cards in September 2013 comprises 284,807 transactions, 492 of which are fraudulent. The sample is tilted, with fraudulent transactions accounting for only 0.172% of total transactions. To protect cardholder privacy, the dataset comprises 31 attributes, 28 obtained by a PCA transformation.

#### 2. Credit card fraud detection dataset 2023

The current study also utilised a different credit card fraud detection from 2023. This collection contains 568,630 operations with 284315 scams [42] user Nelgiriyewithana developed this fresh Kaggle dataset. It purports to include transactions made in 2023 using anonymised European cards to safeguard cardholders’ identities. However, there isn’t much information on the dataset’s quantity, quality, or source.

The article "Anomaly detection in multivariate time series data using deep ensemble models" was retracted in 2025. Reasons: duplicate publication; overlap with earlier publications; suspected computer-generated content; citations of retracted work.

### C. Evaluation of metrics

In this work, these metrics will be evaluated ROC_AUC and PR_AUC. F1, R2 score, ADR, FPR, and accuracy. Precision, also known as specificity, is the proportion of expected class i representatives that accurately categorise. The following formula is used for determining precision:

$$Precision\;Rate=\frac{True\;Positive}{True\;Positive+False\;Positive}$$ (1)

People in class i who are correctly classified are true positives in Eq (1). False positives, on the other hand, are things that have been misclassified and belong to distinct groups.

The recall rate, as sensitivity [43], demonstrates the system’s competency in the model associated with the class of interest, type i. This is how the recall is determined:

$$Recall\;Rate=\frac{True\;Positive}{True\;Positive+False\;Negative}$$ (2)

Bogus negatives are cases that belong in class I but are misclassified in Condition (2).

We process the F-1 score in light of exactness and review conditions (1) and (2). The F-1 score thinks about accuracy and memory balance and gives more unambiguous data on grouping adequacy, for example, unique accuracy and review levels and ideal model assurance. The following is how the F-1 score is evaluated:

$$F-1\;Score=2*\frac{\left(Precision*Recall\right)}{Precision+Recall}$$ (3)

The accuracy indicator is further utilised in assessing achievement [44]. The ratio of accurately detected cases to the absolute number of occurrences is used to calculate accuracy:

$$Accuracy\;Rate=\frac{True\;Positive+True\;Negative}{Total\;Positive+Total\;Negative}$$ (4)

The AUC-ROC curve measures assessment efficiency and considers multiple threshold levels. The AUC (Area Under the Curve) curve is a probability curve that shows how effectively a model can distinguish between distinct groups. On the other hand, the ROC (Receiver Operating Curve) is bent to evaluate class isolation. As a result, the AUC-ROC curve defines a methodology’s ability to distinguish between categories, with a larger AUC indicating greater viability in various types of choosing situations.

The coefficient of connection (R2 score) is a quantitative statistic that indicates how much variation in the dependent variable can be explained by the free variable(s). The model’s all-out fluctuation in the dependent variable is examined to see how effectively the model replicates actual discoveries. R2 values vary from 0 to 1, with higher values indicating a more effective model assault on the data. A score of one implies that the model accurately predicts all of the variability in the dependent variable. A score of 0 shows that the approach does not sufficiently represent the variance of the dependent variable.

The article "Anomaly detection in multivariate time series data using deep ensemble models" was retracted in 2025. Reasons: duplicate publication; overlap with earlier publications; suspected computer-generated content; citations of retracted work.

The MCC measurement considers each of the four components of the disarray lattice (TP, TN, FP, and FN). It is worth between—1 and 1, with 1 being fantastic expectation, 0 addressing irregular expectation, and—1 addressing complete disparity among estimates and realities. It accommodates imbalanced datasets.

The Anomaly Detection Rate (ADR) regarding abnormality discovery addresses the extent of oddities accurately identified by the model. Considering this when evaluating models designed to observe unusual events is critical. The FPR is calculated by dividing the number of inaccurate optimistic estimations by the total number of negatives. It is recorded as FP/(FP + TN) and is especially useful in parallel characterization problems where misleading up-sides should be kept to a minimum.

#### 1. Summary of evaluation metrics

The selection of assessment metrics in this research is highly in line with its aims and the unique characteristics of the problem being addressed. The measures used include accuracy, precision, recall, F1 Score, ROC AUC, PR AUC, MCC, R2 Score, ADR, and FPR. Accuracy assesses the accuracy of the model’s predictions by determining the ratio of predicted adequately to total occurrences. High accuracy suggests a low incidence of false positives, which is critical in anomaly detection to reduce false alarms and guarantee that flagged cases are indeed weird. Recall quantifies the fraction of natural anomalies successfully detected by the model out of all actual anomalies. High recall implies that the model effectively catches most of the anomalies in the dataset, lowering the risk of missing critical anomalies. ROC AUC calculates the trade-off between (TPR or recall) and (FPR) at various threshold values. A greater ROC AUC shows improved discrimination between normal and abnormal cases. PR AUC assesses the trade-off between accuracy and recall at multiple threshold settings. The MCC function balances a model’s performance, especially in binary classification applications such as anomaly detection. In regression problems, the R2 Score indicates the percentage of variation the model explains. ADR calculates the fraction of properly recognized anomalies among all natural anomalies in a dataset. FPR is the fraction of false positives among all cases projected to be anomalous.

These metrics provide a complete picture of a model’s presentation by considering aspects such as exactness, correctness, review, and the tradeoffs between deceptive advantages and fake disadvantages. The specific features and restrictions of the particular situation determine which metric (s) to emphasise.

The article "Anomaly detection in multivariate time series data using deep ensemble models" was retracted in 2025. Reasons: duplicate publication; overlap with earlier publications; suspected computer-generated content; citations of retracted work.

### D. Result and discussion

Deep learning approaches have demonstrated promising results in credit card data processing, with studies identifying irregular transactions, use trends, and merchant transactions utilizing CNN, GNN, DAGMM, Transformer, and LSTM networks. These models are more accurate and sensitive than traditional procedures for detecting anomalies. They may also anticipate future transactions based on expenditure and fraud likelihood, provide accurate estimates, identify probable fraud proactively, optimise fraud detection systems, and improve financial planning.

### E. Comparison of classification result

The experimental results for all classifiers are presented in Table 2, revealing that the chosen classifiers outperform all others in all aspects, as shown in Figs 11–13.

**Fig 11:** CNN-LSTM and their ensembled comparison of classification results on the proposed solution.

**Fig 12:** Transformer-GNN and their ensembled comparison of classification results on proposed.

**Fig 13:** DAGMM comparison of classification results on the proposed solution.

**Table 2:** Comparison of classification results.

Classifier	Dataset	Accuracy	Precision	Recall	F1 Score	ROC AUC	PR AUC	MCC	(R2) Score	ADR	FPR
CNN	Credit Card Fraud Detection	0.9994	0.8181	0.8602	0.8387	0.9299	0.8393	0.8387	0.6685	0.0016	0.8602
LSTM	Credit Card Fraud Detection	0.9994	0.7891	0.8529	0.8197	0.9262	0.8211	0.8201	0.6244	0.0017	0.8529
CNN-LSTM-Ensembled	Credit Card Fraud Detection	0.9994	0.8057	0.8235	0.8145	0.9116	0.8147	0.8142	0.6244	0.0016	0.8235
CNN	Credit Card Fraud Detection 2023	0.9995	0.9996	0.9995	0.9995	0.9995	0.9996	0.9991	0.9983	0.5007	0.9995
LSTM	Credit Card Fraud Detection 2023	0.9996	0.9998	0.9994	0.9996	0.9996	0.9997	0.9992	0.9985	0.5006	0.9994
CNN-LSTM-Ensembled	Credit Card Fraud Detection 2023	0.9997	0.9998	0.9997	0.9997	0.9997	0.9998	0.9995	0.9991	0.5008	0.9997
Transformer	Credit Card Fraud Detection	0.9994	0.8248	0.8308	0.8278	0.9153	0.8279	0.8275	0.6538	0.0016	0.8308
GNN	Credit Card Fraud Detection	0.9994	1.0000	1.0000	0.8413	0.9902	0.8683	0.8410	0.6833	0.0015	1.0000
Transformer-GNN-Ensembled	Credit Card Fraud Detection	0.9994	1.0000	1.0000	0.8436	0.9263	0.8438	0.8434	0.6833	0.0016	0.8529
Transformer	Credit Card Fraud Detection 2023	0.9996	0.9996	0.9996	0.9996	0.9996	0.9997	0.9993	0.9986	0.5008	0.9996
GNN	Credit Card Fraud Detection 2023	0.9996	1.0000	1.0000	0.9996	0.9999	0.9999	0.9993	0.9986	0.5008	1.0000
Transformer-GNN-Ensembled	Credit Card Fraud Detection 2023	0.9996	0.9997	0.9996	0.9996	0.9996	0.9997	0.9993	0.9987	0.5008	0.9996
DAGMM	Credit Card Fraud Detection	0.9704	0.7047	0.7047	0.7047	0.8446	0.8446	0.6892	0.3784	0.0500	0.0155
DAGMM	Credit Card Fraud Detection 2023	0.5185	0.5300	0.0546	0.0991	0.5045	0.5045	0.0208	0.2078	0.0500	0.0455

The article "Anomaly detection in multivariate time series data using deep ensemble models" was retracted in 2025. Reasons: duplicate publication; overlap with earlier publications; suspected computer-generated content; citations of retracted work.

#### 1. CNN

The CNN classifier detected credit card theft on two datasets with an overall accuracy of 99.94%. The model demonstrated a balance of accuracy and recall with a ROC AUC of 92.99% and a PR AUC of 83.93%. When accurate and false positives and negatives were included, the MCC was 83.87%. The R2 score was 66.85%, indicating that the model was well-fitting. The ADR was 0.16%, while the FPR was 0.86%. The model demonstrated accuracy and precision in recognising credit card fraud with a high F1 score, ROC AUC, PR AUC, MCC, and R2 scores. Overall, the CNN classifier proved highly effective in detecting fraudulent transactions.

#### 2. LSTM

The LSTM classifier was employed for credit card fraud detection on two datasets, yielding good accuracy, precision, recall, F1 score, ROC AUC, PR AUC, MCC, R2 score, ADR, and FPR. The model has a 99.94% accuracy rate and a 78.91% false positive rate. The classifier accurately identified 85.29% of positive instances, according to the recall rate of 85.29%. The F1 score was 81.97%, showing that accuracy and recall were balanced. The classifier’s ROC AUC was 92.62%, indicating that it could discriminate among positive and negative categories. The MCC was 82.01% when true and false positives and negatives were combined. The ADR was 0.17%, representing the percentage of accurately detected attacks, while the FPR was 0.85%.

#### 3. CNN-LSTM ensemble

The CNN-LSTM-Ensembled ensemble model, which combines a CNN and an LSTM network, was applied to two credit card fraud detection datasets. The model was 99.94% accurate, with an 80.57% accuracy and an 82.35% recall. The F1 score was 81.45%, with a ROC_AUC of 91.16%. When precision and recall were considered, the PR AUC was 81.47%. The R2 score was 62.44%, while the MCC score was 81.42%. The FPR was 0.84%, while the ADR was 0.16%. When CNN and LSTM models were combined, the ensemble demonstrated outstanding precision, recall, and accuracy, indicating that it may be used to detect fraudulent transactions. The dataset performs admirably, with a minimal false positive rate. Fig 11 depicts the general efficacy of CNN-LSTM and their ensemble.

#### 4. Transformer

Credit card fraud is detected pretty successfully using the Transformer classifier. It has a 99.94% accuracy rate, % precision rate of 82.48%, and % recall rate of 83.08%. The model’s F1 score is 82.78%, and its AUC is 91.53%. The PR AUC is 82.79%, while the MCC is 82.75%. The R2 score is 65.38%, with an attack detection rate of 0.16% and an FPR of 0.84%. The Transformer classifier performed admirably on the Credit Card Fraud Detection 2023 dataset, with a low false positive rate and high AUC values. Its strong F1 score and ROC AUC show that it identifies fraudulent transactions successfully.

The article "Anomaly detection in multivariate time series data using deep ensemble models" was retracted in 2025. Reasons: duplicate publication; overlap with earlier publications; suspected computer-generated content; citations of retracted work.

#### 5. Graph neural networks (GNNs)

When applied to two credit card fraud detection datasets, the Graph Neural Network (GNN) classifier obtained 99.94% accuracy, 100% precision, and 100% recall. The F1 score of 84.13% indicated that accuracy and recall were balanced. The ROC AUC was 99.02%, indicating that the classifier could distinguish between positive and negative categories. When accuracy and recall were considered, the PR AUC was 86.83%. The MCC was 84.10% when true and erroneous positives and negatives were considered. The R2 score was 68.33%, indicating that the model fit the data well. The model performed brilliantly on the Credit Card Fraud Detection 2023 dataset, achieving perfect precision, recall, and accuracy. The model effectively identified fraudulent transactions with a low FPR and excellent AUC values.

#### 6. Transformer-GNN-ensemble

Regarding credit card fraud, the Transformer-GNN-Ensemble model performed exceptionally well, with 99.94% accuracy, precision, and recall of 100%, and F1 and R2 scores of 84.36% and 94.34%, respectively. ROC_AUC, PR_AUC, MCC, ADR, and FPR are 92.63%, 84.38%,.0.16%, and 85.29%, respectively. The model was stable on the 2023 fraud data while retaining high accuracy, recall, and other measures. Its accuracy, precision, and recall on the 2023 dataset are 99.96%, 99.97%, and 99.96%, respectively. Meanwhile, ROC_AUC, PR_AUC, MCC, and FPR have individual values of 99.96%, 99.97%, 99.93%, and 99.96%, respectively. Fig 12 depicts the overall performance of Transformer-GNN and its ensemble on both datasets.

#### 7. Deep autoencoding gaussian mixture model (DAGMM)

In comparison, the DAGMM Model fared significantly worse in detecting credit card fraud, with an accuracy of 97.04%. The model’s accuracy, recall, and F1 score measurements demonstrated a trade-off between detecting fraud and reducing false positives. When applied to the 2023 sample, the DAGMM’s performance dropped drastically, showing potential constraints in responding to emerging fraud tendencies. Fig 13 demonstrates DAGMM’s overall performance on both datasets.

### F. Key findings from the experimental results

Although the CNN, LSTM, CNN-LSTM-Ensemble, Transformer, GNN, and Transformer-GNN-Ensemble models functioned brilliantly over both data sets about precision and accuracy, the DAGMM model showed less flexibility to dynamic fraud patterns. The optimum classifier is decided by the data’s specific requirements and characteristics, with graph-based algorithms proving especially beneficial in finding complex links within credit card transaction data.

The article "Anomaly detection in multivariate time series data using deep ensemble models" was retracted in 2025. Reasons: duplicate publication; overlap with earlier publications; suspected computer-generated content; citations of retracted work.

Furthermore, employing ensemble techniques that combine the capabilities of many models may improve overall performance and resilience in the face of changing fraud environments. Continuous research should focus on scalability and efficiency, particularly in real-time systems, to promptly detect fraudulent transactions.

While the models evaluated demonstrated remarkable capabilities in credit card fraud detection, ongoing research and development are critical to addressing evolving challenges and ensuring the continued effectiveness of fraud detection systems in the dynamic financial transaction landscape. The suggested technique may apply to any time series-related data and activities. This is furthermore effective for stock market forecasting and anomaly detection [45]. This is also significant for forecasting and recognising weather patterns [46]. The intrusion detection challenge [47] needs time series modelling. This may also predict/forecast time series data and discover anomalies. Using many datasets in our study seeks to increase and reinforce the suggested models’ learning capabilities.

The study of anomaly detection using deep ensemble models has critical practical ramifications for many real-world settings, notably in businesses where identifying abnormalities in time series data is vital. These applications include financial transaction fraud detection, network intrusion detection, healthcare monitoring and patient safety, industrial equipment monitoring and predictive maintenance, supply chain management, and energy and grid monitoring. Fraud detection in financial transactions entails finding suspicious patterns and abnormalities in transaction data, allowing financial organisations to detect fraudulent activity in real time and save monetary losses. Network intrusion detection analyses traffic data using deep ensemble models to identify intrusions and cybersecurity risks, improving network security and resilience.

Healthcare monitoring and patient safety entail early identification of vital signs or behaviour abnormalities, which allows for prompt interventions and improves patient outcomes and safety. Industrial equipment monitoring and predictive maintenance can detect abnormalities that indicate a malfunction or impending breakdown early on, allowing for proactive maintenance and reducing downtime costs. In supply chain management, anomaly detection can discover anomalies or disturbances in the flow of products and commodities, allowing for proactive risk management and mitigation. Energy management and grid monitoring can detect abnormalities that indicate energy theft, equipment failure, or system instability, allowing for more efficient energy distribution, fewer blackouts, and increased grid resilience.

The article "Anomaly detection in multivariate time series data using deep ensemble models" was retracted in 2025. Reasons: duplicate publication; overlap with earlier publications; suspected computer-generated content; citations of retracted work.

Finally, the findings of the studies presented in this paper show the promise of deep learning for credit card anomaly identification and forecasting and the necessity for more study in this area. The study findings on anomaly detection using deep ensemble models provide prospects for greater operational efficiency, risk reduction, and enhanced real-time decision-making. Breakthroughs in deep learning algorithms and the increasing availability of annotated data will contribute to future advances in credit card data processing accuracy and efficiency.

## Conclusion

This study looked at deep learning algorithms for time series forecasting and anomaly detection. This research aims to detect anomalies in credit card transactions by employing a range of deep learning methods. According to research, transformers and GNN versions are adequate for these jobs. Furthermore, this study demonstrated that these strategies may successfully achieve sophisticated and indirect patterns in time series data, allowing for better forecasting and outlier detection. The results of these credit card fraud detection approaches demonstrate the efficacy of deep learning models, notably CNN, LSTM, GNN, and their ensembles. These models consistently showed good accuracy, precision, and recall, implying their ability to detect dishonest transactions.

The suggested technique for detecting anomalies using deep ensemble models yields promising results but has significant limits and problems. Data imbalance can result in biased model performance, mitigated by strategies such as oversampling, undersampling, or complex algorithms such as SMOTE. Feature engineering is critical to the success of deep learning models, and poor feature selection or extraction can lead to unsatisfactory performance. Computational resources are a significant barrier, as training deep ensemble models on massive datasets necessitates enormous computational resources. This might include improving model structures, using distributed frameworks, or utilizing cloud computing resources. Model compression approaches can minimize computational burden while maintaining performance. Transfer learning, thorough validation techniques, and robust assessment of varied datasets can all help to increase generalisation to new settings. Hyperparameter tuning, which includes grid search, random search, and Bayesian optimisation, can improve model performance. Data quality and noise can also be enhanced by preprocessing techniques such as noise reduction, outlier identification, and data cleaning. Researchers must overcome these restrictions using methodological advances, algorithmic enhancements, and domain-specific expertise. By carefully evaluating these problems and using relevant solutions, researchers might create more effective anomaly detection methodologies that are more widely applicable and resilient.

The article "Anomaly detection in multivariate time series data using deep ensemble models" was retracted in 2025. Reasons: duplicate publication; overlap with earlier publications; suspected computer-generated content; citations of retracted work.

Lastly, the utility of deep learning models is proved by contrasting multiple classifiers for detecting credit card fraud, specifically CNN networks, LSTM networks, and their ensembles. These models displayed good accuracy, precision, and recall constantly, suggesting their capacity to detect fraudulent transactions while limiting false positives. Furthermore, transformer-based models performed well, demonstrating the versatility of attention approaches while collecting complex data patterns. GNNs (graph neural networks) were also quite successful, mainly when dealing with the complicated links seen in credit card transaction systems. In the future, it will be vital to investigate strategies to increase the adaptability of fraud detection systems to changing patterns. This may require creating models with continuous learning capabilities capable of responding to new fraud tactics. Furthermore, investigating the interpretability of these deep learning models may give valuable insights into the characteristics and relationships underlying their predictions, hence increasing the models’ dependability in real-world applications.
